# Identification of lncRNA Biomarkers and LINC01198 Promotes Progression of Chronic Rhinosinusitis with Nasal Polyps through Sponge miR-6776-5p

This article has been retracted.

**DOI:** 10.1155/2022/9469207

**Published:** 2022-05-06

**Authors:** Xueping Wang, Xiaoyuan Zhu, Li Peng, Yulin Zhao

**Affiliations:** ^1^Department of Otolaryngology Head and Neck Surgery, The First Affiliated Hospital of Zhengzhou University, Zhengzhou, Henan, China 410000; ^2^Department of Obstetrics and Gynecology, The First People's Hospital of Nanyang, Nanyang, Henan, China 473000

## Abstract

**Background:**

Chronic sinusitis (CRS) was a chronic inflammation that originated in the nasal mucosa and affected the health of most people around the world. Chronic rhinosinusitis with nasal polyps (CRSwNP) was one kind of chronic sinusitis. Emerging research had suggested that long noncoding RNAs (lncRNAs) played vital parts in inflammatories and inflammation development.

**Methods:**

We acquired GEO data to analyze the differential expression between the miRNA, immune genes, TF, and lncRNA data in CRSWNP and the corresponding control tissues. Bioinformatic analysis by coexpression of endogenous RNA network and competitive way enrichment, analysis, and forecasting functions of these noncoding RNA. The different pathway expressions in CRSwNP patients were confirmed using GSVA to analyze the differentially expressed immune genes and TF data sets in CRSwNP patients. The differential immune gene and transcription factor data set in CRSwNP perform functional notes and protein-protein interaction (PPI) network structure. We predicted the potential genes and RNAs related to CRSWNP by constructing a ceRNA network. In addition, we also used 19 hub immune genes to predict the potential drugs of CRSWNP. lncRNA biomarkers in CRSwNP were identified by lncRNAs LASSO regression. The CIBERSORT algorithm was used to contrast the divergence in immune infiltrations between CRSwNP and usual inferior turbinate organizations in 22 immunocyte subgroups.

**Results:**

We identified a total of 48 miRNAs, 304 lncRNAs, 92 TFs, and 525 immune genes as CRSwNP-specific RNAs. GO and KEGG pathways both analyzed differentially expressed immune genes and transcription factor data sets. We predicted the potential genes GNG7, TUSC8, LINC01198, and has-miR-6776-5p by constructing ceRNA and PPI networks. At the same time, we found that the above genes were involved in two important pathways: chemokine signal path and PI3K/AKT signal path. In addition, we predicted 5 small molecule drugs to treat CRSwNP by analyzing 19 central immune genes, namely, danazol, ikarugamycin, semustine, cefamandole, and molindone. Finally, we identified 5 biomarkers in CRSwNP, namely, LINC01198, LINC01094, LINC01798, LINC01829, and LINC01320.

**Conclusions:**

We had identified CRSwNP-related miRNAs, lncRNAs, TFs, and immune genes, which may be making use of latent therapeutic target for CRSwNP. At the same time, we identified 5 lncRNA biomarkers in CRSwNP. The results of this study showed that LINC01198 promoted the progression of CRSwNPs through spongy miR-6776-5p. Our studies provide a new way for further analyses of the pathogenesis of CRSwNP.

## 1. Background

Chronic sinusitis (CRS) was a chronic inflammation that comes of the mucosa of the sneezers and affects the physique of many person on a global scale [1, 2]. On the basis of epidemiological datas, CRS affected 10.9% and 7. 0% of the number of people in Europe and South Korea, separately [3, 4]. Chronic rhinosinusitis with nasal polyps (CRSwNP) was a clinical manifestation of chronic sinusitis. CRS patients mainly had the following symptoms: nasal congestion, hyposmia, olfactory asthenia, encephalalgias, facial pain, or pressure, of which CRSwNP and nasal congestion and anosmia are related [5–7]. According to clinical data, CRSwNP patients were prone to drug resistance during treatment, so patients with CRSwNP were often difficult to cure. At the same time, the studies had found that the incidence of CRSwNP had nothing to do with whether the patient had undergone repeated sinus surgery and the expression level of local corticosteroids or long-term systemic glucocorticoids [8, 9]. To make a long story short, pursuing the latent mechanism of CRSwNP is significant for the cure of CRSwNP.

Long noncoding RNAs (lncRNAs) were long, exceed 200 nucleotides, and referred to RNA that could not encode protein [10]. More and more studies had proved that lncRNAs participated in almost all parts of gene control, consisting of epigenetic developmental control, nucleocytoplasmic transship, and transcription [11]. Therefore, lncRNAs affect most cell biological proceeding consisting of cell growth, proliferation, metastasis, invasion, and divergence [11, 12]. Abnormal lncRNA expression was a common feature of many diseases [13]. However, there were few studies on CRSwNP and lncRNAs. As a specific differentiated lncRNA, LINC01198, a contraction of long intergenic nonprotein coding RNA 1198, was located on chromosome 13 and initially captured in a glioma study where LINC01198 was predicted to be remarkably associated with tumor grade and overall prognosis on clinical tissue level by virtue of bioinformatic data analysis, preliminarily implying the oncogenic nature of it. The latest research has suggested that the abnormal expression of LINC01198 was related to glioma and rectal cancer. It was relevant to the incidence and progression of bladder cancer [14–16]. However, the role of LNC01198 in other inflammatory diseases was not reported.

MicroRNAs (miRNAs) were small, 20-24 nucleotides, and were newly discovered type of noncoding RNAs that mediated protein levels by binding target mRNAs. It belongs to endogenous RNA. At present, some studies had demonstrated that miRNAs played a crucial role in the occurrence and progression of cancer [17]. Studies had found that some miRNAs were differentially expressed in CRSwNP and affected its development [8, 18]. The effect of miR-6776-5p has already been evidenced by current studies, such as promoting the occurrence of renal cancer development by inhibiting the degradation of oncogene TRPM3 [19]. Both microRNAs and lncRNAs played important roles in regulating gene expression and involved a variety of biological processes. Salmena et al. proposed a hypothesis about competitive endogenous RNA (Cerna) in 2011 and proved it [20–22]. The ceRNA referred to the existence of certain RNAs (herein referred to as ceRNAs) and targeted miRNAs that had a common binding site and a competitive activity, thereby affecting the function of the target miRNA. The ceRNAs could interact with the target miRNA to control transcription group expression [23].

In this study, we identified 5 lncRNA biomarkers in CRSwNP (LINC01198, LINC01094, LINC01798, LINC01829, and LINC01320). We found that compared with the control group, LINC01198 was downregulated in CRSwNP. We established a ceRNA network and found that LINC01198, TUSC8, miR-6776-5p, and GNG7 had a mutual regulatory relationship. At the same time, they were related to the PI3K/AKT signaling pathway. We speculated that LINC01198 could regulate miR-6776-5p through ceRNA and might promote the proceeding of CRSwNPs through the PI3K/AKT signaling pathway. Therefore, LINC01198 may be a latent target for the cure of CRSwNP. In addition, we also enriched the immune gene GNG7 in CRSwNP with GSEA and predicted the results of the small molecule drug treatment of 19 hub immune genes for CRSwNP. Finally, we found that the M2 macrophages between the resting dendritic cells in CRSwNP may be synergistic by immunopermeation analysis. The research results obtained from this article are very important and can supply a novel thinking model for prevention, cure, and prognosis of CRSwNP.

## 2. Materials and Methods

### 2.1. GEO Data Set Collection

We retrieved the microarray data sets (mRNA and lncRNA) from the GEO database (http://www.ncbi.nlm.nih.gov/geo) through R GEOquery package. The data set accession numbers used are GSE136825, GSE36830, and GSE169376.

### 2.2. Record Pretreatment and Abnormal Expression Analysis

The crude TXT data gathered from the GEO database was pretreated using the microarray data (limma) R package. Batch effects were adjusted by the combat function of sva package of R software using empirical Bayes frameworks after merging all microarray data. Finally, the expression values were normalized according to the normalizeBetweenArrays function of the package of limma in R software so that the expression values have similar distribution across a set of arrays. For the obtained limma, the explored sequence was downloaded from the explanatory note platform and justified with the human-genome to obtain the expression level of miRNA. We used the R limma package to detect differential expression of the miRNA data set GSE169376. We used ∣logFC | >1 and FDR < 0.05 as the filter strip to the final differentially expressed miRNA, immune gene, TF (transcription factors), and lncRNA. They were named as DmiRNA, DimGene, DTFgene, and DlncRNA data sets. As a result, R ggplot2 package was used to paint the volcano map and the heat map.

### 2.3. Target Prediction and Functional Enrichment

All predicted targets were subjected to Gene Ontology (https://www.kegg.jp/) analysis and genome KEGG (https://www.kegg.jp) type pathway enrichment analysis, which was implemented by the R package clusterProfilter [24, 25] (*P* < 0.01).

### 2.4. GSVA Analysis

Gene set variation analysis (GSVA), a functional enrichment analysis method similar to gene set enrichment analysis (GSEA), allowed the assessment of underlying pathway activity variation in each sample by preinputting a selected gene set. It can draw such a conclusion that as an uncommon method, GSVA may have amazing latent capacity in related research of signal path.

GSVA was used to distinguish signal path levels among CRSwNP patients. GSVA had a capacity to compute enrichment scores of selected gene sets for every patient. Therefore, through GSVA, the patients' gene set matrix including path enrichment score was obtained.

### 2.5. PPI Network Construction

The PPI network was drawn from the String database (https://www.string-db.org/) against the differential immune gene and transcription factor data set in CRSwNP, and the parameter setting was confidence > 0.9. We used the clusterProfiler gene to enrich the KEGG pathway and combined with PPI network to draw TF-immune genes-pathway network through Cytoscape 3.8.0.

We used the online database search tool String to build the PPI network and DTFgene network and score the fusion ≥ 0.9 as the critical point ≥ 0.9 and removed the protein nodes that cannot interacted with the other. In addition, we used Cytoscape (version: 3.8.0) to analyze the PPI network to screen the caused modules and hub genes. The MCODE (version: 2.0.0) plug-in was used to choose the significant clustering module according to the standard MCODE score > 10 and the amount of nodes > 20 and used the cluster preliquid to carry out the path enrichment analysis package of the genes in these modules. Then, using the apoptosis (version: 0.1) insert to show the PPI network, genes with a degree > 10 were identified as hub genes in CRSwNP.

### 2.6. ceRNA Network Construction

We used TargetScan, miRDB, and miRanda online tools to reversely predict miRNA for 9 hub immune genes, took the intersection to obtain miRNA, and then took the intersection with DmiRNA. We used lncbase (https://diana.e-ce.uth. gr/lncbasev3/) and MiRcode (http://www.mircode.org/) to forecast the relationship between lncRNAs and miRNAs and obtain miRNA target lncRNA by taking the intersection and then took the intersection with DlncRNA. According to the lncRNA-miRNA-mRNA ceRNA regulation principle, lncRNA and miRNA were negatively correlated, lncRNA and mRNA were positively correlated, and miRNAs and mRNAs were negatively correlated. lncRNA-miRNA-mRNA ceRNA regulation relationship Tab. was screened out. Finally, we merged the hub TF-immune genes-pathway network to carry out the lncRNA-miRNA-TF-immune gene-pathway ceRNA network, visualized the network through Cytoscape, and constructed the key immune gene lncRNA-miRNA-Hub gene-pathway ceRNA network.

### 2.7. Statistical Analysis

Statistical analysis was implemented using R 3.6.3. digital datas, which were certified to obey a normal distribution shown as the mean ± standard, and the differences between means were analyzed using Student's *t*-test. ANOVA analysis was used to predict lncRNA, immune genes, TF, and miRNA abnormal expression among diverse groups. The considerably lncRNA, immune genes, TF, and miRNA were inquired into limma R package. A threshold value of∣log2FC | ≥1andFDR < 0.05, the heat mapping were showed form ggplot 2, ComplexHeatmap.

## 3. Results

### 3.1. Identification of Differentially Expressed miRNA, Immune Genes, TF, and lncRNA in CRSWNP

We used the GEO database to analyze differential expression of the substance of miRNA, lncRNA, TF (transcription factors), and immune gene in CRSwNP, and the results were displayed in a volcano graph. Compared with the control group, a total of 48 lower miRNAs were abnormally expressed in CRSwNP. 12 raised miRNAs and 36 miRNAs were appraised between CRSwNP and control (Figure 1(a)). There were 304 abnormally expressed lncRNAs, 141 were upregulated and 163 reduced, that were identified between CRSwNP and control (Figure 1(b)). There were 92 abnormally expressed TFs, among 44 were raised and 48 were downregulated (Figure 1(c)). There were 525 abnormally expressed immune genes, of which 394 were upregulated and 131 downregulated (Figure 1(d)). We performed a 2D hierarchical clustering analysis on the above data. The results are shown in Figure 2, revealing the differences in the expression profiles of CRSwNP miRNA, lncRNA, TF (transcription factors), and immune gene (∣logFC | >1 and FDR < 0.05). The specific data set is shown in Table 1.

### 3.2. Functional Annotation of Gene Enrichment and Prediction Targets

We implemented functional enrichment of the abnormally expressed immune genes and transcription factor data sets in CRSwNP. Through KEGG and GO enrichment analysis, we discovered that the above genes are significantly enriched in the following three types of functions, including biological processes (BP), cellular fraction (CC), and molecular function (MF). The top 10 enrichment terms in BP, CC, and MF are provided in Figure 3(a). In Figure 3(b), KEGG analysis appraised 30 paths in total, several of which interact with cytokine-cytokine receptors, neuroactive ligand-receptor interaction, PI3K-Akt signal path, chemokine signal path, and calcium. The above results revealed that these pathways are involved in the pathological progress of CRSwNP. We used the GSVA method to calculate the standardized pathway enrichment scores of 658 immune gene set-based pathways for each CRSwNP patient using the CRSwNP immunization and TF data sets, shown in the heat map (Figures 3(c) and 3(d)). We found that in some CRSwNP patients, the pathway enrichment scores based on CRSwNP immunization and TF collection seemed to be partially aggregated. Many patients had dependently high path enrichment fractions, while others could not spread higher expression models. This indicated that CRSwNP patients had different pathway expression profiles, which was consistent with some published studies.  Table 2 is the description of the related terms of the KEGG pathway.  Table 3 is the specific data of the KEGG pathway GSVA analysis.

### 3.3. PPI Network Establisher and Hub Gene Authentication

We are grateful for the suggestion. To be more clear and in accordance with the reviewer concerns, we have revised the manuscript accordingly. “We used the clusterProfiler gene to enrich the KEGG pathway and combined it with the PPI network and used Cytoscape version 3.8.0 to draw the TF-immune genes-pathway network (Figure 4(b)). We used Cytoscape MCODE plug-in (version: 2.0.0) and CytoHubba plug-in (version: 0.1) to screen out hub network and hub genes (Figures 4(c) and 4(d)).

### 3.4. Construction of ceRNA Network on Account of Differential DmiRNA, DimGene, DTFgene, and DlncRNA

We established ceRNA network on account of expression profiles of DmiRNA, DimGene, DTFgene, DlncRNA, and CRSwNP patients. We used hub immune genes to reversely predict miRNAs, then intersected with differentially expressed miRNAs, and obtained 14 miRNA nodes (8 upregulation and 6 downregulation). We used lncbase and MiRcode to forecast the relationship between lncRNAs and miRNAs and took the intersection to obtain 38 lncRNA nodes (20 upregulated and 18 downregulated). The result is shown in Figure 5(a) (∣logFC | >1 and FDR < 0.05). According to the establishment of the lncRNA-miRNA-mRNA ceRNA regulatory relationship list in CRSwNP (Table 4). We merged the hub TF-immune genes-pathway network to carry out the lncRNA-miRNA-TF-immune gene-pathway ceRNA network, visualized the network through Cytoscape, and constructed the key immune gene lncRNA-miRNA-Hub gene-pathway ceRNA network, and the obtained two important pathways are shown in Figure 5(b).

### 3.5. CMAP: Small Molecule Therapeutic Drugs

The enrichment outcomes of PIK3R1 revealed that it was significantly enriched in the JAK-STAT signal path, T Toll-like receptor signal path, TNF signal path, fluid shear pressure, and atheromatosis AGE-RAGE signal path in diabetes mellitus difficult problem and chemokine signaling pathway (Figure 6(a)). Using the CMAP database, we used 19 hub immune genes (KMT2A, PTPN1, TFAP2C, TLR7, SMARCE1, KLRD1, LIFR, FZD1, FST, TGFB2, KLRC4, CYSLTR1, PIK3R1, BCAR1, TRIM36, CCR9, THBS1, NOD2, and C7) to forecast latent therapeutic medicines for CRSWNP. Five drugs in total, called danazol, ikarugamycin, semustine, cefamandole, and molindone, were identified (Figures 6(b) and 6(c)). Hub immune genes were used to forecast latent medicines for the cure of CRSwNP .

### 3.6. Construction of CRSWNP Diagnostic Model Based on Immune-Related Genes

LASSO coefficient profiles of 42 lncRNAs are displayed in Figure 7(a), and the line of dashes make known the selected value by tenfold cross-validation. Tenfold cross-proving for harmonious parameter choice in the LASSO pattern is displayed in Figure 7(b). In Figures 7(a) and 7(b), the quantity above the chart delegates the quantity of paths related in the LASSO pattern. Through the LASSO regression process, 5 of 42 lncRNA set were filtered for subsequent analysis (Table 5). ROC were painted and their AUCs decided to appraise the diagnostic value of the key lncRNAs using the pROC package in R 3.6.3. DlncRNAs have an AUC of >0.85 and were differentially regulated. Data sets were used to establish one binomial LASSO pattern deal with R. In the training and validation set, 50% of specimens in the GSE169376 data set was stochastic choice by the caret package in R 3.6.3 (Figures 7(c) and 7(d) ). As *λ* raises, LASSO prefers decrease the regression coefficient to zero. lncRNA with AUC > 0.85 in the GSE169376 data sets was defined as biomark lncRNAs (Figure 7(e)). The expression levels of 5 lncRNA biomarkers in CRSwNP patients and normal controls are shown (Figures 7(f)–7(j)).

### 3.7. Immune Infiltration Analyses

Due to technical limitations, CRSwNP immune penetration has not been fully revealed, especially in subgroups with low cell numbers. Using the CIBERSORT algorithm, we first investigated the differences in immune infiltration between 42 CRSwNP and 28 normal inferior turbinate tissues in 22 immune cell parts.  Figure 8(a) reveals the scale of immune cells in 28 normal controls and 42 CRSwNP patients. Obviously, plasma cells and B cell naive were explained for the most permeating cells, notably in 28 normal control tissues, but M2 macrophages were increased in CRSwNP tissue. The abnormal expression ratio of immune permeating cells in CRSwNP is displayed in Figure 8(b). Only M2 macrophages, T cell CD8, and plasma cells were abnormally expressed, and M2 macrophages were increased in CRSwNP tissue (*P* values, 0.001). Plasma cells and T cell CD8 were downregulated in CRSwNP tissue, and the *P* values of the two types of immune cells were 0.048 and 0.044. From CRSwNPA (Figure 8(c)), the ratio of immune cells in 42 CRSwNP and 28 normal controls did not show significant population bias aggregation but individual differences.  Figure 8(d) shows the relevance between abnormally expression forms of immune cells. M2 macrophages were actively bound up with dendritic cells resting (*r* = 0.33) and passively bound up with B cell naive. Macrophages M0, Macrophages M1, T cells, CD4 memory resting, Plasma cells (*r* = −0.4,*r* = −0.32,*r* = −0.21,*r* = −0.22and*r* = −0.39, respectively). M2 macrophages between dendritic cell resting in CRSwNP may be synergistic. However, it is indicated that the function of B cell naive, macrophage M0, macrophage M1, T cell CD4 memory resting, and plasma cells in CRSwNP was antagonistic (Figures 8(e)–8(j)).

The overall design idea of the experiment is shown in Figure 9.

## 4. Discussion

In our research, we found a ceRNA regulatory network and a PPI network in CRSwNP and identified five lncRNA biomarkers. Among them, LINC01094 and LINC01320 were upregulated in CRSwNP, while LINC01798, LINC01198, and LINC01829 were downregulated. We combined the ceRNA network and the PPI network to find that TUSC8 and LINC01198 coregulate miR-6776-5p and then regulated the chemokine signal path and PI3K/Akt signal path through GNG7 to act a major part in the development of CRSwNP.

CRSwNP was a clinical manifestation of chronic sinusitis [26]. CRSwNP involved the mucosa of the sinuses, which was a common chronic inflammatory disease. The molecular mechanism of its pathogenicity remained unclear. Therefore, identifying new biomarkers, strengthening predictions, and understanding the underlying mechanisms were essential for the treatment of CRSwNP. The causes and progression of CRSwNP were the combined results of many factors, such as genetic disorders and pathological factors. In European and American Caucasians, more than 80% of CRSwNP have characteristic eosinophil infiltration, dominated by T helper 2 cell (Th2 cell) type inflammation [27, 28]. However, in yellow Asians, there is more infiltration of neutrophils and other inflammatory cells, with T helper 1 cell (Thl cell) or T Helper 17 cell (Th L7 cell) as the dominant type of inflammation. So, we have reason to believe that eosinophils and helper T cells are the key cells in its pathogenesis [27, 28]. At the molecular level, CRSwNP may be caused by abnormalities in multiple noncoding RNAs, transcription factors, and immune genes [29–32]. As new noncoding RNAs, lncRNAs played vital parts in the progress of CRSwNP. For instance, lncRNA XLOC_010280 came to light to affect the development of eosinophilic inflammation by influencing CCL18 [33]. There were many pathological features of CRSwNP, including infiltration of inflammatory cells and interstitial edema [34]. Both this research and previous studies indicated that the pathogenic factors of CRSwNP may be related to abnormal expression of noncoding RNAs and immune dysregulation, despite the mechanisms were still unknown [35]. For instance, Ma et al. found that the inflammatory response regulator LRRK2 was highly expressed in patients with CRSwNP and was positively correlated with CD3 expression. At the same time, they also found that IL-17A can raise LRRK2 and inhibit the level of noncoding RNA NRON, thereby promoting the development of CRSwNP [36]. Interestingly, relative evidence suggested that both increased mucus secretion and macrophage activation were related to the pathogenesis of CRSwNP, indicating that immune infiltration analysis could be used to determine the risk of CRSwNP [35]. However, the pathogenesis of CRSwNP was affected by environmental factors and the underlying mechanism was still largely unknown. Therefore, our investigation of abnormally altered genes will help to understand the pathogenesis of CRSwNP.

At present, large-scale RNA sequencing had determined more than 10,000 lncRNAs in mammalian genomes including humans. More and more researches had affirmed that lncRNAs and miRNAs acted a vital part in most cell biological proceedings containing cell growth, proliferation, invasion, invasion, and cytodifferentiation [37, 38]. Abnormal expression of lncRNAs and miRNAs was a common feature of the pathogenesis of many diseases [39, 40]. For example, the study by Wang et al. showed that by constructing a ceRNA network of miRNAs and lncRNAs, it came to light that the etiopathogenesis of CRSwNP was related to AGR2, FAM3D, PIP, TMC, and DSE [29, 33]. In addition, the study found that lncRNA was related to the pathological development of CRSwNP-sinusitis with rhinopolyps and asthma type 2 hyperinflammation, and determined the expression profile of lncRNA in CRSwNP [29, 33]. Zhang et al. [41] have found that lncRNA GATA3-AS1 is specifically expressed in Th2 cells and lncRNA GATA3-AS1 and GATA3 genes are regulated by the same transcriptional regulatory element, which may play an important role in Th2L-type immune response. Zhu et al. [42] showed that the expression of LNC-GAS5 was upregulated in exosomes in nasal mucus of patients with allergic rhinitis and in exosomes of human nasal epithelial cells stimulated by ovalbumin. LNC-GAS5 inhibits the differentiation of Th1 cells by downregulating T-BET and EZH2 and promotes the differentiation of Th2 cells by upregulating GATA-3, suggesting that LNC-GAS5 is a key mediator of Th1/Th2 differentiation. In addition, Yue et al. [43] found that LNC-000632 expression was downregulated in nasal mucosal samples from patients with allergic rhinitis and IL-13-stimulated nasal epithelial cells. LNC-000632 targets MIR-498 and inhibits IL-13-induced production of granulocyte-macrophage colony stimulating factor, eosinophil chemokine, and MUAC5AC. But the above study results were confined only to the relevance between miRNAs and lncRNAs in CRSwNP. In our research, we carried on a genome expression profile both in CRSwNP and homologous control groups. We appraised and analyzed abnormally expressed miRNA, immune genes, TF, and lncRNA to illustrate the etiopathogenesis of CRSwNP. Our research found that a gross of 48 miRNAs, 304 lncRNAs, 92 TFs, and 525 immune genes was unusually expressed in CRSwNP. As far as we know, this is the first to systematically identify and analyze noncoding RNA, TFs, and immune genes related to CRSwNP.

Our research found that the pathological progress of CRSwNP was related to cytokine-cytokine receptor interaction, neuroactive ligand-receptor interaction, PI3K-Akt signal path, chemokine signal path, and calcium. In addition, we found that in some CRSwNP patients, immune genes were based on abnormal expression of CRSwNP and pathway enrichment collected by TF overlap, which was the same as previous studies. Therefore, we judged that cell proliferation and immune regulation were also involved in the pathogenesis of CRSwNP. Based on the above analysis, we further used the String database to draw a PPI network for the differential immune gene and transcription factor data set in CRSwNP. We established a ceRNA network on account of the expression profiles of DmiRNA, DimGene, DTFgene, DlncRNA, and CRSwNP patients. We got 14 miRNA nodes (8 upregulated and 6 downregulated) and 38 lncRNA nodes (20 upregulated and 18 downregulated). Based on the above analysis, we further selected a pair of Cernas: TUSC8/LINC01198/has-miR-6776-5p/GNG7.

As a member of lncRNA family, LINC01198 was identified in tumor cells. In latest studies, it had been put forward that LINC01198-originated chromosome 13 could affect many biological functions. For instance, LINC01198 adjusted multiplication in various diseases and cancers [44, 45]. In the light of S. Chen et al., LINC01198 was bound up with cell apoptosis [15]. Sun et al. suggested that LINC01198 played a regulatory role in the biological function of bladder cancer [16]. Base on the above, it could be verdicted that LINC01198 had to do with the effect of pathological process in CRSwNP. To verify that the effect of LINC01198 on CRSwNP may be adjusted by expression, we quantified the expression of LINC01198 in CRSwNP and control and proved that LINC01198 was downregulated in CRSwNP, which indicated that the low expression of LINC01198 promoted the pathogenesis of CRSwNP. miRNA imbalance was bound up with diversified inflammations and unusual immune responses, such as pulmonary fibrosis and asthma. Fundamentally, present studies had confirmed that assorted miRNAs were abnormally expressed in CRSwNP and impacted the progress of CRSwNP inflammation [46, 47]. Zhong et al. identified that miR-6776-5p was linked to calcification of vascular smooth muscle cells induced by high glucose/senescence [48]. On the basis of Li et al., miR-6776-5p was bound up with the invasions of renal cell cancer via restraining TRPM3 [19]. Our study corroborated that miR-6776-5p was upregulated in CRSwNP patients. Its high expression in CRSwNP tissue makes it clear that it may be relevant to the occurrence of CRSwNP. We discovered that LINC01198 promoted CRSwNP by meditating miR-6776-5p, but this still requires test verification.

A variety of lncRNAs were abnormally expressed in CRSwNP and were related to the occurrence of CRSwNP. Despite these lncRNAs were not proposed in this research, they may be related to the differences between different detection platforms [30, 49–51]. For example, it had been reported that AKT1, CDH1, PIK3R1, CBL, LRP1, MALAT1, and XIST had been shown to be involved in the pathogenesis of CRSWNP [52]. Draw ROC map according to LASSO model, and choose DlncRNA with AUC > 0.85 and differentially expressed as lncRNA biomarkers. From this, we identified LINC01198, LINC01094, LINC01798, LINC01829, and LINC01320 as CRSWNP biomarkers. The above evidence indicated that our results provided new data for CRSwNP biomarkers. However, these data still need to be experimentally verified.

According to the literature, the inflammatory mechanism in CRSwNP may be related to TH2 polarization and tissue eosinophils [53, 54]. We collected data on 22 immune cell subsets in 42 CRSwNP and 28 normal inferior turbinate tissues. Through immune penetration analysis, we found that there was a positive correlation between M2 macrophages and resting dendritic cells in CRSwNP. However, a negative correlation with B cell naiveness, macrophage M0, macrophage M1, T cells, and plasma cells. This indicated that there may be a synergistic effect between M2 macrophages and dendritic cells in CRSwNP, while CRSwNP had antagonistic effects on B cell naiveness, macrophage M0, macrophage M1, T cell CD4 memory cessation, and plasma cell function. These results indicated that immune disorders were related to the pathogenesis of CRSwNP, but this result had individual differences. In addition, in order to find effective medicines for the remedy of CRSwNP, we used the CMAP database to detect 19 immune genes and identified 5 drugs, namely, danazol, idarubicin, semustine, cephalosporin, and morpholinone.

Importantly, known, abnormally expressed lncRNAs and miRNAs can regulate the pathological process of many diseases including CRSwNP. According to the establishment of a ceRNA network, we found that there may be mutual regulation between LINC01198, TUSC8, miR-6776-5p, and GNG7 that were abnormally expressed in CRSwNP. In addition, they were related to the PI3K/AKT signal path. This may involve a critical mechanism in CRSwNP. Further research on these RNAs may announce more significant message about the pathogenesis of CRSwNP.

## 5. Conclusion

We constructed a ceRNA network specific to CRSwNP related to immune gene, TF, miRNA, and lncRNA and identified 5 lncRNA biomarkers. We found that LINC01198, TUSC8, miR-6776-5p, and GNG7 were among the ceRNA networks. There was a mutual regulatory relationship related to the PI3K/AKT signal path. This research may provide a new idea for further understanding of the pathogenesis of this disease.

## Figures and Tables

**Figure 1:** Volcano plots of abnormally expressed miRNA, immune genes, TF, and lncRNA in CRSwNP. Volcano plots of abnormally expressed miRNA (a), immune genes (b), TF, and lncRNA in CRSwNP and normal. Red and green points correspond to log2FC (∣log2FC | >0.5) up/down, respectively, and indicate FDR < 0.05. (a–d). Volcano plot of differential expression of miRNA (a), immune genes (b), transcription factors (c), and lncRNA (d) with log (fold change) as the abscissa and -log10 (*P* value) as the ordinate. Red and green splashes represent the genes that were significantly up- or downregulated in CRSwNP, respectively. Green splashes mean genes without significantly different expression. FDR < 0.05 and ∣logFC | >0.5.

**Figure 2:** The heat map of abnormally expressed miRNA, immune genes, TF, and lncRNA in normal and CRSwNP. The heat map of abnormally expressed miRNA, immune genes, TF, and lncRNA in normal and CRSwNP hierarchically clustered. Each list indicates a sample and every line indicates an miRNA (a), immune gene (b), transcription factors (c), and lncRNA (d). The expression value for each line was normalized by the *z*-score. Red indicates high relative expression and green indicates low relative expression (∣logFC | >1 and FDR < 0.05).

**Figure 3:** The enrichment of differentially expressed immune genes and transcription factors predicted targets in CRSwNP. Used to visualize the enrichment of differentially expressed immune genes and transcription factor prediction targets in CRSwNP. Detailed GO enrichment and KEGG information are presented in the bubble map. Gene Ontology (GO) Kyoto Encyclopedia of Genes and Genomes (KEGG) pathological analysis of immune and TF genes. Significantly enriched pathways featured *P* < 0.001. The analysis was conducted using R clusterProfilter. (a) GO enrichment analyses of TF and immune genes. *y*-axis represents GO terms, and *x*-axis represents GeneRatio. The number of genes enriched in the enrichment term is indicated by the size of the node. The importance of the GO term is indicated by the color, and the red indicates the highest significance. (b) KEGG pathway enrichment analyses of TF and immune genes. The *y*-axis represents the KEGG term. The *x*-axis represents GeneRatio. The number of genes enriched in the enrichment term is represented by the size of the node. The importance of the KEGG term is represented by color, and red represents the highest significance. (c) The heat map of differentially expressed immune genes for KEGG pathway horizontally represents KEGG terminology; longitudinal direction means sample, red means upregulation, and green means downregulation. (d) The heat map of differentially expressed immune genes for GO; horizontal means GO term, longitudinal means sample, red means upregulation, and green means downregulation.

**Figure 4:** Construction of TF-immune genes-pathway networks. (a) The protein-protein interaction (PPI) network. (b) TF-immune genes-pathway network. (c) The hub network by MCODE. (d) The hub network by CytoHubba.

**Figure 5:** The results of using mRNA to stepwise reverse predict miRNA and lncRNA and constructing a ceRNA network. (a) The flow chart of predicted miRNA target gene and network construction. (b) The hub lncRNA-miRNA-mRNA ceRNA pathway.

**Figure 6:** Predictive results of small molecule drug therapy for CRSwNP. Single-gene GSEA enrichment results of GNG7 gene and prediction results of potential small molecule drugs for the treatment of CRSwNP based on 19 hub immune genes. (a) lncRNA-miRNA-pathway ceRNA network. (b) Single-gene enrichment analysis of GNG7 gene (GSEA, gene set enrichment analysis). (c) Prediction results of targeted drugs.

**Figure 7:** Development and validation of lncRNA biomarkers. (a) The LASSO regression. (b) LASSO coefficient profiles of the 5 lncRNAs. (c) Receiver operating characteristic (ROC) curve of the CRSWNP for the training set (GSE136825). (d) Receiver operating characteristic (ROC) curve of the CRSWNP for validation set (GSE136825). (e) Receiver operating characteristic (ROC) curve of the CRSWNP for external data set (GSE36830). The *x*-axis represents the 1-specificity and *y*-axis represents the sensitivity. AUC: area under the curve. (f) Gene expression levels of LINC01198. (g) Gene expression levels of LINC01094. (h) Gene expression levels of LINC01798. (i) Gene expression levels of LINC01829. (j) Gene expression levels of LINC01320.

**Figure 8:** Visualization of immune cell infiltration and correlation between GNG7, TUSC8, and LINC01198 expressions and infiltrating immune cells. (a) The composition of infiltrating immune cells. (b) Violin plot of differences of immune cell infiltration. (c) Principal component analysis cluster plot of immune cell infiltration. (d) Correlation matrix of proportions of 22 types of infiltrating immune cells. (e) Correlation between GNG7 expression and plasma cells (*R* = 0.56, *p* = 4e − 07). (f) Correlation between LINC01198 expression and plasma cells (*R* = 0.21, *p* = 0.077). (g) Correlation between TUSC8 expression and plasma cells (*R* = 0.33, *p* = 0.0053). (h) Correlation between GNG7 expression and macrophage M2 (*R* = −0.33, *p* = 0.0055). (i) Correlation between LINC01198 expression and macrophage M2 (*R* = −0.16, *p* = 0.17). (j) Correlation between TUSC8 expression and macrophage M2 (*R* = −0.35, *p* = 0.0037).

**Figure 9:** Flow chart.

**Table 1:** GEO data set.

GEO accession	Platforms	Normal	Case	Organism	Experiment type
GSE136825	GPL20301	28	42	Homo sapiens	Expression profiling by array
GSE36830	GPL570	6	12	Homo sapiens	Expression profiling by array
GSE169376	GPL21572	3	3	Homo sapiens	Noncoding RNA profiling by array

**Table 2:** Kyoto Encyclopedia of Genes and Genomes (KEGG) pathway.

#term ID	Term description	False discovery rate
hsa04060	Cytokine-cytokine receptor interaction	3.30E-28
hsa05150	Staphylococcus aureus infection	7.73E-15
hsa04062	Chemokine signaling pathway	9.22E-15
hsa04380	Osteoclast differentiation	2.36E-10
hsa04610	Complement and coagulation cascades	1.91E-09
hsa04630	Jak-STAT signaling pathway	2.83E-09
hsa04659	Th17 cell differentiation	6.15E-08
hsa05200	Pathways in cancer	1.43E-07
hsa05202	Transcriptional misregulation in cancer	1.43E-07
hsa05133	Pertussis	1.93E-07
hsa04145	Phagosome	2.19E-07
hsa04657	IL-17 signaling pathway	3.48E-07
hsa04640	Hematopoietic cell lineage	2.41E-06
hsa05152	Tuberculosis	2.41E-06
hsa04151	PI3K-Akt signaling pathway	2.84E-06
hsa05140	Leishmaniasis	2.97E-06
hsa05323	Rheumatoid arthritis	3.09E-06
hsa05322	Systematic lupus erythematosus	9.88-06
hsa04668	TNF signaling pathway	4.13E-05
hsa05221	Acute myeloid leukemia	5.32E-05
hsa04650	Natural killer cell mediated cytotoxicity	0.00016
hsa05321	Inflammatory bowel disease (IBD)	0.00017
hsa04015	Rap1 signaling pathway	0.00019
hsa04621	NOD-like receptor signaling pathway	0.00021
hsa05142	Chagas disease (American trypanosomiasis)	0.00035
hsa04658	Th1 and Th2 cell differentiation	0.00047
hsa04672	Intestinal immune network for IgA production	0.00047
hsa05167	Kaposi's sarcoma-associated herpesvirus infection	0.00054
hsa05215	Prostate cancer	0.00091
hsa05418	Fluid shear stress and atherosclerosis	0.00091

**Table 3:** GSVA analysis of KEGG pathway.

ID	logFC	*P* value	Adj. *P* value
KEGG_PURINE_METABOLISM	-0.68	1.50E-15	6.46E-14
KEGG_TGF_BETA_SIGNALING_PATHWAY	-0.63	7.20E-14	2.81E-12
KEGG_VASCULAR_SMOOTH_MUSCLE_CONTRACTION	0.57	8.01E-16	3.52E-14
KEGG_ALZHEIMERS_DISEASE	-0.56	1.36E-13	5.17E-12
KEGG_DILATED_CARDIOMYOPATHY	-0.40	1.70E-09	5.10E-08
KEGG_INSULIN_SIGNALING_PATHWAY	-0.36	2.04E-10	7.35E-09
KEGG_HYPERTROPHIC_CARDIOMYOPATHY_HCM	-0.33	1.68E-06	4.20E-05
KEGG_GAP_JUNCTION	-0.28	2.80E-08	7.83E-07
KEGG_CALCIUM_SIGNALING_PATHWAY	-0.27	1.36E-07	3.67E-06
KEGG_MELANOGENESIS	-0.24	3.21E-06	7.70E-05
KEGG_PROSTATE_CANCER	-0.21	0.000136386	0.002591328
KEGG_CHEMOKINE_SIGNALING_PATHWAY	0.22	0.000230059	0.003910995
KEGG_CYTOKINE_CYTOKINE_RECEPTOR_INTERACTION	0.23	1.19E-05	0.000261605
KEGG_AXON_GUIDANCE	0.26	7.29E-05	0.001457423
KEGG_INTESTINAL_IMMUNE_NETWORK_FOR_IGA_PRODUCTION	0.32	2.82E-05	0.000591205
KEGG_NOD_LIKE_RECEPTOR_SIGNALING_PATHWAY	0.37	6.28E-06	0.000144332
KEGG_HEMATOPOIETIC_CELL_LINEAGE	0.38	1.88E-07	4.90E-06
KEGG_JAK_STAT_SIGNALING_PATHWAY	0.39	8.90E-09	2.58E-07
KEGG_CELL_CYCLE	0.39	0.000147908	0.002662341
KEGG_ENDOCYTOSIS	0.43	1.63E-15	6.85E-14
KEGG_COMPLEMENT_AND_COAGULATION_CASCADES	0.46	6.72E-10	2.15E-08
KEGG_TOLL_LIKE_RECEPTOR_SIGNALING PATHWAY	0.52	2.06E-10	7.35E-09
KEGG_LEUKOCYTE_TRANSENDOTHELIAL_MIGRATION	0.55	1.12E-14	4.59E-13
KEGG_SYSTEMATIC_LUPUS_ERYTHEMATOSUS	0.57	2.20E-10	7.49E-09
KEGG_NATURAL_KILLER_CELL_MEDIATED_CYTOTOXICITY	0.63	1.67E-12	6.18E-11
KEGG_T_CELL_RECEPTOR_SIGNALING_PATHWAY	0.63	1.29E-09	3.99E-08
KEGG_LEISHMANIA_INFECTION	0.64	1.29E-14	5.16E-13
KEGG_FC_GAMMA_R_MEDIATED_PHAGOCYTOSIS	0.67	2.35E-10	7.77E-09

**Table 4:** lncRNA-miRNA-mRNA ceRNA regulatory relationship list.

lncRNA	logFC	Mature miRNA	logFC	Immune gene	logFC
TUSC8	-2.566634992	hsa-miR-6776-5p	1.849653653	GNG7	-1.236759067
LINC01198	-3.423148908	hsa-miR-6776-5p	1.849653653	GNG7	-1.236759067

**Table 5:** Multi-Cox analysis of lncRNA showed 5 lncRNA with a biomark.

lncRNA	Coef	HR	HR. 95L	HR. 95H	Cox *P* value
LINC01094	0.001471451	1.001472534	1.000057684	1.002889385	0.041357096
LINC01798	0.079829794	1.83102701	1.017376455	1.53075104	0.12443396
LINC01829	0.126665257	1.35037009	1.009532575	1.276144072	0.034119673
LINC01320	0.063348029	1.065397564	0.992187746	1.144009261	0.081152175
LINC01998	0.186665257	0.977302291	0.947132838	1.008432744	0.002443396

## Data Availability

The data used to support the findings of this study are included within the article.
